The article "Effects of All-Inclusive and Hierarchical Rehabilitation Nursing Model Combined with Acupuncture on Limb Function and Quality of Life in Elderly Patients with Cerebral Infarction during Convalescence" was published in 2022. Journal: J Healthc Eng.

# Effects of All-Inclusive and Hierarchical Rehabilitation Nursing Model Combined with Acupuncture on Limb Function and Quality of Life in Elderly Patients with Cerebral Infarction during Convalescence

**DOI:** 10.1155/2022/2654729

**Published:** 2022-04-13

**Authors:** Lan Zuo, Mingzi Sun

**Affiliations:** ^1^Department of Nursing, Affiliated Hospital of Inner Mongolia Chifeng University, Chifeng 024099, Inner Mongolia, China; ^2^Department of Rehabilitation Physiotherapy, Affiliated Hospital of Inner Mongolia Chifeng University, Chifeng 024099, Inner Mongolia, China

## Abstract

**Objective:**

To investigate effects of all-inclusive and hierarchical rehabilitation nursing model combined with acupuncture on limb function and quality of life in elderly patients with cerebral infarction during convalescence.

**Methods:**

Eighty elderly patients with cerebral infarction who were treated in our hospital (February 2018–February 2020) and met the inclusion and exclusion criteria were chosen as the research objects, and their materials were analyzed in the way of retrospective study. They were equably randomized into observation group and reference group. Based on the acupuncture treatment, the patients in the observation group and the reference group were given routine rehabilitation nursing and all-inclusive and hierarchical rehabilitation nursing respectively for three months. The simplified Fugl-Meyer Assessment (FMA) scores, Modified Edinburgh-Scandinavian Stroke Scale (MESSS) scores, Activities of Daily Living Scale (ADL) scores, and Stroke-Specific Quality of Life Scale (SS-QOL) scores in the two groups before and after intervention were recorded, and the changes of limb function, neurological function, and living quality of the patients in the two groups were analyzed.

**Results:**

Compared with the reference group, the observation group after intervention achieved prominently higher FMA score (*P* < 0.001), markedly lower MESSS score (*P* < 0.001), and signally higher SS-QOL scores (*P* < 0.05). After intervention, the observation group achieved obviously higher ADL score than the reference group (68.88 ± 8.91 vs 59.00 ± 8.38, *P* < 0.001).

**Conclusion:**

The all-inclusive and hierarchical rehabilitation nursing model combined with acupuncture can accelerate the recovery of neurological function of the elderly patients with cerebral infarction, enhance the rehabilitation of their limb function, and markedly improve their quality of life. Therefore, this model has referential significance in clinic.

## 1. Introduction

Cerebral infarction, also known as cerebral arterial thrombosis, mostly occurs in middle-aged and elderly people, and its main physiological and pathological process is that the patients suffer from ischemic-hypoxic necrosis of local cerebral tissues on the basis of atherosclerosis and successive neurological impairment and deficit [1]. According to the epidemiological survey data of stroke in 2013, the incidence and mortality of cerebral infarction in China were much higher than the world average level, and its incidence reached up to 42% among Chinese men and 37% among Chinese women [2]. In 2019, the *Lancet* further confirmed that the cerebral stroke was the primary cause of death in China from 1990 to 2017 [3]. Moreover, the mortality and disability rates of elderly patients are much higher than those of the young- and middle-aged patients, because the elderly patients have decreased physical function and are complicated with various underlying diseases [4, 5]. Nowadays, as the population aging intensifies in China, the patients suffering from cerebral infarction are increasing. Although its mortality has decreased compared with a decade ago, its disability rate remains high [6]. About 75.0% of the patients living with the disease are disabled due to neurological deficit, and 40.0% are severely disabled [7, 8]. The patients' daily life is severely impacted. According to the study of Okuda et al., the limb dysfunction and failure of independent living enhance the negative emotions of the elderly patients with cerebral infarction and significantly decrease their living wills [9]. Therefore, it is extremely important to improve the patients' physical function and quality of life.

The article "Effects of All-Inclusive and Hierarchical Rehabilitation Nursing Model Combined with Acupuncture on Limb Function and Quality of Life in Elderly Patients with Cerebral Infarction during Convalescence" was published in 2022. Journal: J Healthc Eng.

At present, the 1 year after the onset of cerebral infarction is referred to as the convalescence, during which the symptom control in the patients is effective and scientific rehabilitation intervention can improve their neurological function and enhance their motor ability [10]. The practice has shown that the effect of joint rehabilitation intervention of traditional Chinese medicine (TCM) and Western medicine during convalescence is better than that of Western medicine alone. Acupuncture, as a common rehabilitation method for cerebral infarction in TCM, effectively promotes the flow of qi and blood, sharpens mind, and resuscitates the brain. Due to the poor psychological and physical status and unsatisfactory treatment compliance of the elderly patients, it is necessary to simultaneously provide them with all-inclusive rehabilitation nursing and good treatment conditions in clinic. In recent years, some studies have shown that the hierarchical rehabilitation nursing model can balance the contradictions between nursing services and professional development, because there are great differences in the experience and technological level of the nursing staff with different ranks, and the hierarchical rehabilitation nursing provides the patients with more considerable and complete nursing services and is conducive to improving the quality of clinical nursing [11]. At present, no study has applied the hierarchical rehabilitation nursing model in the nursing of elderly patients with cerebral infarction. This paper investigates the effects of all-inclusive and hierarchical rehabilitation nursing model combined with acupuncture on limb function and quality of life in elderly patients with cerebral infarction, summarized as follows.

The article "Effects of All-Inclusive and Hierarchical Rehabilitation Nursing Model Combined with Acupuncture on Limb Function and Quality of Life in Elderly Patients with Cerebral Infarction during Convalescence" was published in 2022. Journal: J Healthc Eng.

## 2. Materials and Methods

### 2.1. Inclusion Criteria

(1) The patients were diagnosed to be cerebral infarction by magnetic resonance imaging (MRI) and brain computed tomography (CT) and met the diagnostic criteria for cerebral infarction formulated by World Health Organization (WHO) [12]. (2) The patients were above 60 years old. (3) The patients had clear mind and no cognitive dysfunction, and they could cooperate the researchers well to complete the study. (4) The patients had stable life signs and conditions.

### 2.2. Exclusion Criteria

(1) The patients were unconscious or had mental illness and could not communicate with others. (2) The patients were complicated with severe diabetes or hypertension. (3) The patients had secondary cerebral hemorrhage, dysfunction of important organs, hematopoietic dysfunction, active bleeding, or malignant tumor. (4) The patients could not coordinate with the study.

### 2.3. Clinical Data

According to the inclusion and exclusion criteria, 80 elderly patients with cerebral infarction treated in our hospital (February 2018–February 2020) were brought into the study, and all the patients had signed the informed consent. This study was conducted under the guidance of the Declaration of Helsinki (2013) [13]. The 80 patients were equably randomized into observation group and reference group, with 40 patients in each group. In the observation group, there were 28 males and 12 females with a mean age of (72.30 ± 7.13) years old. The patients' average height was (164.32 ± 6.67) cm, their mean body mass was (60.32 ± 5.20) kg, their mean infarct size was (1.65 ± 0.54) cm, and their mean course of disease was (6.32 ± 0.62) months. Besides, there were 15 cases with lacuna infarction, 6 cases with temporal lobe infarction, 15 cases with basal ganglia cerebral infarction, and 4 cases with cerebral infarction in the parietal lobe. In the reference group, there were 26 males and 14 females with a mean age of (72.35 ± 5.95) years old. The patients' average height was (164.81 ± 7.57) cm, their mean body mass was (60.45 ± 5.23) kg, their mean infarct size was (1.62 ± 0.50) cm, and their mean course of disease was (6.35 ± 0.65) months. Besides, there were 16 cases with lacuna infarction, 5 cases with temporal lobe infarction, 14 cases with basal ganglia cerebral infarction, and 5 cases with cerebral infarction in the parietal lobe. No significant difference in the patients' age, sex ratio, infarct size, infarction location, and other general data between the two groups was observed (*P* > 0.05), and the patients in the two groups could be taken as the study samples.

The article "Effects of All-Inclusive and Hierarchical Rehabilitation Nursing Model Combined with Acupuncture on Limb Function and Quality of Life in Elderly Patients with Cerebral Infarction during Convalescence" was published in 2022. Journal: J Healthc Eng.

### 2.4. Methods

#### 2.4.1. Acupuncture Treatment

All the patients were given routine drug treatment in neurological department and consciousness-restoring resuscitation (Xingnao Kaiqiao) acupuncture. The patients were given acupuncture at the acupoints of Renzhong, Sanyinjiao, Neiguan, Jiquan, Chize, and Weizhong. The needles were inserted with diagonal stabbing and reducing method at the acupoint of Renzhong, with diagonal stabbing and reinforcing method at the acupoint of Sanyinjiao, with straight needling and reducing method at the acupoints of Neiguan, Jiquan, Chize, and Weizhong. The needles were retained at each acupoint for 30 min after the arrival of qi, 1 time/d, and 6 d/week. Six days were a course of treatment, and the patients took a day off before receiving the next course. The acupuncture treatment lasted for 3 months.

#### 2.4.2. Reference Group

The reference group was given routine rehabilitation nursing on the basis of acupuncture treatment. The nursing staff assist the patients with rehabilitation training by giving them drug use and diet guidance, movement guidance (including standing, squatting, and sitting movement), and posture nursing.

#### 2.4.3. Observation Group

The observation group received all-inclusive and hierarchical rehabilitation nursing on the basis of acupuncture, and the specific steps were as follows. (1) Establishing the rehabilitation nursing teams. The team members were divided into 3 grades, including responsible team leaders, primary nurses, and assistant nurses. The responsible team leaders were the charge nurses or vice-director nurses with more than 10 years of nursing experience, the primary nurses were the nurses with 5–10 years of nursing experience, and the assistant nurses were the nurses with less than 5 years of nursing experience. All team members reviewed related literature on hierarchical nursing and learned from advanced experience in the manner of evidence-based nursing. In addition, the responsibility of each grade was specified according to the characteristics of the patients with cerebral infarction in our hospital, so as to clarify the individual responsibility. (2) Establishing the shift system. The nurses of different grades were divided into 3 nursing groups according to their educational level, specialized level, communication ability, and other factors. The 8-hour continuous shift system was implemented, and the team leaders needed to communicate with the nurses and coordinate the scheduling to ensure the integrity and continuity of the rehabilitation nursing. (3) Training. The training contents, mainly including relevant systems, nursing knowledge and professional skills about the rehabilitation nursing of the patients with cerebral infarction, were arranged in accordance with the rehabilitation nursing requirements of each grade, so as to improve the nursing staff's ability of individualized analysis and judgment of the patients' clinical symptoms, monitoring parameters, and nursing key points. (4) Division of work. ① Assistant nurses were mainly responsible for the patients' basic nursing, such as morning and evening nursing, ward ventilation, and bedding changing, and they should improve the quality of basic nursing to provide the patients with good conditions of recovery. ② Primary nurses were mainly responsible for the patients' routine nursing, such as injection and puncture, and they should improve the eligible rate of the routine nursing operation to ensure the effective progression of the routine nursing. ③ The charge nurses were in charge of the patients with cerebral infarction in all respects, including the health education, mental nursing, recovery guidance, and management of daily life. The elderly patients with cerebral infarction were more likely to develop such adverse emotions as anxiety and irritability due to the disease factors, which affected their compliance with the rehabilitation nursing. Therefore, the charge nurses need to carefully observe the patients' emotional changes and solve their psychological problems in time to ensure that the patients kept good psychological states and received the rehabilitation nursing with positive and healthy attitudes. The charge nurses provided guidance on the patients' simple activities in their daily lives and rehabilitation training in standing or walking according to the patients' conditions, regularly checked the patients' physical conditions, and formulated targeted nutritious diets to strengthen their body immunity. The elderly patients with cerebral infarction stayed in bed for a long time, so they had difficulty in turning over and were likely to be complicated with dermatosis, such as pressure ulcer. Hence, the charge nurses needed to offer the patients posture nursing and tried to keep them in lying position on the health side. When the patients took lying position on the affected side, the charge nurses should help the patients to turn over to avoid pressure ulcer and other complications. After the patients being admitted, their affected limbs were wiped with warm water every day, and they were given the massage with 50% alcohol before going to bed at night to prevent their joints from deforming and being stiff. ④ The vice-director nurses were mainly responsible for the patients' rehabilitation training and difficult nursing operations. After the patients' signs stabilized, the reasonable, scientific, and efficient rehabilitation plans were formulated on the basis of their conditions, and the patients were informed of relevant matters needing attention and methods of rehabilitation training to enhance their cooperation. Then, the rehabilitation training was conducted, and the patients were instructed to move limbs while lying in bed, like stretching out the hands and bending the elbows. After the patients could get out of bed, they did standing balance exercise, torsion training, Tai Chi, and other daily training with the help of vice-director nurses. The nurses should control the intensity of activities, follow the principle of gradual improvement, and timely adjust rehabilitation plans according to the patients' recovery. The vice-director nurses should encourage the patients to read books, listen to music, and watch TV, because proper sensory stimulation was conducive to improving the patients' language sensibility and speeding up the recovery of neurological function. The vice-director nurses could massage the patients' upper limbs with kneading method and lower limbs with rolling method. The massage strength should be from light to stronger and the patients' reaction should be observed.

The article "Effects of All-Inclusive and Hierarchical Rehabilitation Nursing Model Combined with Acupuncture on Limb Function and Quality of Life in Elderly Patients with Cerebral Infarction during Convalescence" was published in 2022. Journal: J Healthc Eng.

### 2.5. Observational Criteria

#### 2.5.1. FMA

Fugl-Meyer Assessment (FMA) [14] was used to assess the patients' limb function before and after intervention. The patients sit when taking the assessment of upper limb function, including reflex activity, associated movements of flexor muscles and extensor muscles, other activities accompanied with associated movement, separatist movement, normal reflection activity, wrist stability, flexion and extension of the fingers, and coordination and finger-to-nose test. When taking the assessment of lower limb function, the patients took the supine, sitting, and standing positions. When taking the supine position, the patients were tested the reflex activity, associated movement of flexor muscles, and coordination/speed. When taking the sitting position, they were tested associated movements and normal reflection activity. When taking the standing position, they were tested separatist movement. The total score of this scale was 100 points, with 66 points in the upper limb function and 34 points in the lower limb function. Higher scores indicated lighter motor dysfunction.

#### 2.5.2. MESSS

Modified Edinburgh-Scandinavian Stroke Scale (MESSS) [15] was used to assess the recovery of neurological function before and after intervention. At first, the patients' consciousness (maximal stimulus and optimum reaction) was assessed. If the patients were unable to answer the questions correctly, the examinations of fist clenching and extension and eye opening and closing were conducted. Those who were unable to complete the above examination further received the examination of limb function, including strong local stimulation to the diseased limb, horizontal gaze, facial paralysis, speech, and upper limb muscle strength. The total score of the scale was 45 points, and higher scores indicated severer damage of advanced central nervous system.

#### 2.5.3. ADL

Activities of Daily Living Scale (ADL) [16] were adopted to assess the patients' abilities of activities daily living before and after intervention. This scale included the assessment of eating, bathing, making-up and washing, dressing, stool control, urine control, going to toilet, bed-chair transfer, walking on level ground, and stairs-climbing, with three evaluation levels of 0 point, 5 points, and 10 points for each item. The total score of this scale was 100 points, and higher scores indicated better abilities of activities of daily living.

#### 2.5.4. SS-QOL

The Stroke-Specific Quality of Life Scale (SS-QOL) [17] was used to evaluate the patients' quality of life before and after intervention. This scale included 12 evaluation dimensions of energy (15 points), family roles (15 points), language (25 points), mobility (30 points), mood (25 points), personality (15 points), self-care (25 points), social roles (25 points), thinking (15 points), upper extremity function (25 points), vision (15 points), and work/productivity (15 points). The total score of this scale was 245 points. Higher scores indicated better quality of life.

### 2.6. Statistical Treatment

This study adopted SPSS20.0 as the data processing software and GraphPad Prism 7 (GraphPad Software, San Diego, USA) as the graph drawing software. The study included count data and measurement data and used X^2^ test and *t* test. When *P* < 0.05, the differences were considered statistically significant.

## 3. Results

### 3.1. FMA

Compared with the reference group, the observation group achieved prominently higher FMA score after intervention (*P* < 0.001; Figure 1).

The article "Effects of All-Inclusive and Hierarchical Rehabilitation Nursing Model Combined with Acupuncture on Limb Function and Quality of Life in Elderly Patients with Cerebral Infarction during Convalescence" was published in 2022. Journal: J Healthc Eng.

No prominent difference in the FMA score of upper limbs between the two groups before intervention was found (29.50 ± 3.75 vs 29.50 ± 3.33, *P* > 0.05). Compared with the reference group, the observation group had prominently higher FMA score of upper limbs after intervention (52.85 ± 4.70 vs 44.68 ± 4.81, *P* < 0.001).

No obvious difference in the FMA score of lower limbs between the two groups before intervention was found (14.60 ± 3.22 vs 14.60 ± 3.18, *P* > 0.05). Compared with the reference group, the observation group had markedly higher FMA score of lower limbs after intervention (27.00 ± 3.54 vs 21.40 ± 3.27, *P* < 0.001).

### 3.2. MESSS

No prominent difference in the MESSS score between the two groups before intervention was found (22.10 ± 2.18 vs 22.13 ± 2.18, *P* > 0.05). Compared with the reference group, the observation group had much lower MESSS score after intervention (14.28 ± 1.64 vs 18.10 ± 1.62, *P* < 0.001).

### 3.3. ADL

No remarkable difference in the ADL score between the two groups before intervention was found (37.50 ± 8.29 vs 37.63 ± 9.01, *P* > 0.05). Compared with the reference group, the observation group had markedly higher ADL score after intervention (68.88 ± 8.91 vs 59.00 ± 8.38, *P* < 0.001).

### 3.4. SS-QOL

Compared with the reference group, the observation group achieved much higher SS-QOL scores after intervention (*P* < 0.05; Table 1).

## 4. Discussion

The incidence and development of cerebral infarction are closely related to thrombosis and atherosclerosis plaque rupture. The pathophysiology changes cause damages to the neurological function and affect the normal control of nervous system over the motor function of limbs. Conducting rehabilitation intervention within 1 year after the onset of cerebral infarction can relieve the patients' neurological impairment, accelerate the recovery of their limb motor function, and improve their quality of life [18]. However, although the common Western medicine intervention has positive effects on patients with cerebral infarction during convalescence, it cannot effectively control the disease progression and cannot significantly improve the patients' limb movement function and quality of life [19]. In addition, scholars Wild et al. have found that basic Western medicine intervention takes effect slowly, and the prolonged rehabilitation intervention may result in the loss of patients' confidence in the treatment, which is not conducive to maintaining their treatment compliance [20]. Because the elderly patients are often complicated with multiple underlying diseases and have limited ability of daily activities, the scientific and efficient intervention during convalescence is the key to ensuring their health psychology and improving their treatment compliance. The studies in recent years have shown that the combination of TCM and Western medicine can accelerate the neurological recovery. According to TCM, cerebral infarction belongs to the category of “apoplexy” and is usually caused by qi stagnation and blood stasis, so the treatment for it should focus on promoting qi to activate blood, so as to relieve the phlegm-blood stasis and obstruction of meridians and alleviate the disturbance of consciousness and clumsy physical activities [21]. Acupuncture is a common TCM intervention, and the acupoints in this study can cooperate with each other to regulate yin and yang, and the patients' neurological functions were recovered to some level and their limb functions were improved after the acupuncture.

The article "Effects of All-Inclusive and Hierarchical Rehabilitation Nursing Model Combined with Acupuncture on Limb Function and Quality of Life in Elderly Patients with Cerebral Infarction during Convalescence" was published in 2022. Journal: J Healthc Eng.

Compared with the reference group, the patients in the observation group had better rehabilitation efficacy in neurological and limb function, because the observation group received efficient nursing intervention on the basis of acupuncture. At this stage, the nursing intervention commonly used in clinics during convalescence mainly aims at the patients' limb rehabilitation, relieving their clinical symptoms and recovering their living ability. Although such nursing intervention has certain effects, it ignores the patients' subjective initiative. Indeed, it does not take the patients with cerebral infarction as the center of rehabilitation nursing [22]. Although the recovery of limb function is the goal of rehabilitation nursing, it is not the sole focus of the rehabilitation, and the main focus is the patient. The study of Liu et al. has further indicated that the effect of routine nursing in balancing the nursing resources is not satisfactory, and the nursing staff with different ranks and professional levels did not fully play their values, causing a waste of nursing resources to a certain extent [23]. Compared with the routine nursing, hierarchical nursing better meets the clinical needs of the patients with cerebral infarction. For example, the nurses may slightly lack theoretical knowledge and clinical experience, so they are mainly responsible for the patients' basic nursing [24], which is conducive to providing punctual and efficient basic nursing. The senior nurses already possess the knowledge base and practical operation ability, so they can take charge of the patients' routine nursing and provide good conditions for the patients to speed up their recovery. The charge nurses are the primary nurses in charge of the patients with cerebral infarction and provide them with all-round services since their admission, which can effectively improve the “disease-centered” nursing model [25], reduce the negative psychology of the elderly patients with cerebral infarction, and improve their satisfaction with the nursing and cooperation with the rehabilitation nursing. With the joint efforts of the nurses, the patients generally develop positive psychology and the condition for physical rehabilitation, based on which the vice-director nurses can provide rehabilitation guidance according to the patients' actual conditions, so as to fully improve the quality of rehabilitation nursing and optimize the effect of rehabilitation nursing. Therefore, the observation group had better neurological function and limb motor function after intervention compared with the reference group (*P* < 0.001); after intervention, the observation group achieved obviously higher ADL score than the reference group (68.88 ± 8.91 vs 59.00 ± 8.38, *P* < 0.001); the patients in the observation group had higher living wills and better quality of life. In the long term, the all-inclusive and hierarchical rehabilitation nursing model can effectively reduce the incidence of nurse-patient disputes. This study provides more reference for reducing the medical burden of cerebral infarction in China.

The article "Effects of All-Inclusive and Hierarchical Rehabilitation Nursing Model Combined with Acupuncture on Limb Function and Quality of Life in Elderly Patients with Cerebral Infarction during Convalescence" was published in 2022. Journal: J Healthc Eng.

At present, the mainstream rehabilitation nursing still has some deficiencies, impeding tit from exerting maximum efficacy, so it is urgently needed to be improved. The all-inclusive and hierarchical rehabilitation nursing model combined with acupuncture can accelerate the recovery of neurological function of the elderly patients with cerebral infarction, enhance the rehabilitation of their limb function, and markedly improve their quality of life. Therefore, this model has referential significance in clinics.

## Figures and Tables

**Figure 1:** Comparison of FMA scores ($\bar{x}$ ± *s*, points). (a) The scores of upper limb function and (b) the scores of lower limb function .

**Table 1:** Comparison of SS-QOL scores ($\bar{x}$ ± *s*, points).

Group	Observation group	Reference group	*t*	*P* value
*Before intervention*				
Energy	4.63 ± 0.58	4.60 ± 0.54	0.239	0.811
Family roles	6.10 ± 0.62	6.10 ± 0.66	0.000	1.000
Language	8.23 ± 1.54	8.20 ± 1.42	0.091	0.928
Mobility	9.18 ± 0.67	9.18 ± 0.70	0.000	1.000
Mood	6.05 ± 0.55	6.08 ± 0.72	0.209	0.835
Personality	4.85 ± 0.73	4.75 ± 0.70	0.625	0.534
Self-care	6.93 ± 0.65	6.90 ± 1.04	0.155	0.878
Social roles	6.33 ± 0.52	6.30 ± 0.46	0.273	0.785
Thinking	5.10 ± 0.62	5.00 ± 0.59	0.739	0.462
Upper extremity function	6.88 ± 1.05	6.83 ± 1.09	0.209	0.835
Vision	7.03 ± 0.72	6.98 ± 1.15	0.233	0.816
Work/productivity	5.13 ± 0.56	5.10 ± 0.73	0.206	0.837
*After intervention*				
Energy	5.98 ± 1.39	5.35 ± 0.73	2.538	0.013
Family roles	7.38 ± 1.49	6.45 ± 0.77	3.507	0.001
Language	9.85 ± 2.13	8.73 ± 1.40	2.779	0.007
Mobility	16.33 ± 3.41	13.15 ± 1.80	5.216	<0.001
Mood	8.18 ± 1.38	7.28 ± 1.20	3.113	0.003
Personality	6.03 ± 1.29	5.10 ± 0.77	3.915	<0.001
Self-care	11.45 ± 2.69	10.23 ± 2.04	2.285	0.025
Social roles	8.48 ± 1.53	7.73 ± 0.16	3.083	0.003
Thinking	6.43 ± 1.16	5.48 ± 0.74	4.367	<0.001
Upper extremity function	11.43 ± 1.58	10.05 ± 1.75	3.702	<0.001
Vision	8.05 ± 1.07	7.28 ± 0.87	3.531	0.001
Work/productivity	6.18 ± 0.77	5.40 ± 0.73	4.649	<0.001

The article "Effects of All-Inclusive and Hierarchical Rehabilitation Nursing Model Combined with Acupuncture on Limb Function and Quality of Life in Elderly Patients with Cerebral Infarction during Convalescence" was published in 2022. Journal: J Healthc Eng.

## Data Availability

Data that support the findings of this study are available on reasonable request from the corresponding author.

## References

[1] Cong X. F., Liu S. B., Ma J. X., Wang W. J., Chen B., Li J. H. (2021). [Association between self-rated health status and risk of stroke in Chinese adults: a prospective study]. *Zhonghua Liuxingbingxue Zazhi*.

[2] Hirayama K., Fuchigami T., Morioka S. (2021). Transcranial direct electrical stimulation for hand function in a stroke patient with severe upper limb paralysis due to lenticulostriate artery occlusion: a case report. *Journal of Medical Case Reports*.

[3] Willer Alexandra K., Jürgen H., Anita T. (2021). Women with cerebral infarction feature worse clinical profiles at admission but comparable success to men during long-term inpatient neurorehabilitation. *Frontiers in Aging Neuroscience*.

[4] Jia L. Y., Du Y.-H. (2021). [Electroacupuncture of “Shuigou”(GV26) improves neurological function by promoting angioge-nesis and Shh signaling in ischemic cerebral tissue of rats with cerebral infarction]. *Zhen Ci Yan Jiu*.

[5] Yao L. L., Yuan S., Wu Z. N. (2022). Contralateral S1 function is involved in electroacupuncture treatment-mediated recovery after focal unilateral M1 infarction. *Neural regeneration research*.

[6] Yan B., Zhang H., Liu J. (2021). Application of quantitative CT imaging in rehabilitation nursing of cerebral apoplexy patients. *Pakistan journal of medical sciences*.

[7] Xu T. Q., Lin W. Z., Feng Y. L. (2022). Leukoaraiosis is associated with clinical symptom severity, poor neurological function prognosis and stroke recurrence in mild intracerebral hemorrhage: a prospective multi-center cohort study. *Neural regeneration research*.

[8] Sui Y. F., Tong L. Q., Zhang X. Y., Song Z. H., Guo T. C. (2021). Effects of paired associated stimulation with different stimulation position on motor cortex excitability and upper limb motor function in patients with cerebral infarction. *Journal of Clinical Neuroscience: Official Journal of the Neurosurgical Society of Australasia*.

The article "Effects of All-Inclusive and Hierarchical Rehabilitation Nursing Model Combined with Acupuncture on Limb Function and Quality of Life in Elderly Patients with Cerebral Infarction during Convalescence" was published in 2022. Journal: J Healthc Eng.

[9] Okuda Y., Aoike F., Shiraishi S. (2021). Functional recoveries of patients with branch atheromatous disease after rehabilitation: Comparison with other types of cerebral infarction and importance of stratification by clinical categories. *Restorative Neurology and Neuroscience*.

[10] Chen Y. C., Tsai S. J. (2021). Bilateral cerebral infarction in diabetic ketoacidosis and bilateral internal carotid artery occlusion: a case report and review of literature. *World journal of clinical cases*.

[11] Zhang Z. H., Zhang X.-C., Guang-Xia N. (2021). [Thrombolysis combined with acupuncture therapy for acute cerebral infarction: a Meta-analysis of randomized controlled trials]. *Zhen Ci Yan Jiu*.

[12] Wang L., Shan M. (2021). Effects of empathy nursing on the quality of life and treatment compliance of elderly patients with cerebral infarction. *American Journal of Tourism Research*.

[13] World Medical Association (2013). World Medical Association Declaration of Helsinki: ethical principles for medical research involving human subjects. *JAMA*.

[14] Li Z., Shang N., Fan G., Li M., Zang Z. (2021). Effect of nursing based on the hopeless self-esteem theory plus multi-dimensional intensive nursing for elderly patients with acute cerebral infarction complicated with depression. *American Journal of Tourism Research*.

[15] Lykov Y. A., Mikryukov A. V., Chefranova Z. Y., Yatsenko E. A., Vlasov P. N. (2020). Improving the diagnosis, treatment and secondary prevention of stroke using a unified online system: primary vascular department - regional vascular center - family doctor. *Zhurnal nevrologii i psikhiatrii im. S.S. Korsakova*.

[16] Cao D., Chu N., Yu H., Sun M. (2021). Role of comprehensive nursing care in improving the prognosis and mood of patients with secondary cerebral infarction after craniocerebral injury. *American Journal of Tourism Research*.

[17] Zeng J., Chen F., Chen Y. (2021). Predictors of hemorrhagic complications after intravenous thrombolysis in acute cerebral infarction patients. *Medicine*.

[18] An X., Zeng L., Shen L., Jiang Y. (2021). Influences of a hierarchical nursing model on rescue outcomes and nursing quality of patients with acute cerebral infarction. *American Journal of Tourism Research*.

[19] Liao Y., Ye T., Liang S. (2021). Clinical nursing pathway improves disease cognition and quality of life of elderly patients with hypertension and cerebral infarction. *Am J Transl Res*.

[20] Wild B., Heider D., Böhlen F., Schöttker B., Muhlack D. C., König H.-H., Slaets J. (2019). Caring for the elderly: a person-centered segmentation approach for exploring the association between health care needs, mental health care use, and costs in Germany. *PLoS One*.

The article "Effects of All-Inclusive and Hierarchical Rehabilitation Nursing Model Combined with Acupuncture on Limb Function and Quality of Life in Elderly Patients with Cerebral Infarction during Convalescence" was published in 2022. Journal: J Healthc Eng.

[21] Chang M. C., Park S. W., Lee B.-J., Park D. (2020). Relationship between recovery of motor function and neuropsychological functioning in cerebral infarction patients: the importance of social functioning in motor recovery. *Journal of Integrative Neuroscience*.

[22] Wang J., Ran C., Pan P., Wang Y., Zhao Y. (2021). Rehabilitation training combined acupuncture for limb hemiplegia caused by cerebral infarction. *Medicine*.

[23] Liu Y., Qu M., Wang N., Wang L. (2021). Effects of an evidence-based nursing intervention on neurological function and serum inflammatory cytokines in patients with acute cerebral infarction: a randomized controlled trial. *Restorative Neurology and Neuroscience*.

[24] Wang Y., Xing J., Zhang R. (2021). Effect and safety of acupuncture on cerebrovascular reserve in patients with acute cerebral infarction. *Medicine*.

[25] Han H., Xin L., Jiang H. N., Ke X., Ying W. (2021). [Effect of early acupuncture on cognitive function in patients with vascular dementia after cerebral infarction]. *Zhongguo Zhen Jiu*.

